# Intravenous Drip of Somatostatin Followed by Restricted Fluid Resuscitation to Treat Upper Gastrointestinal Bleeding in Patients with Liver Cirrhosis

**DOI:** 10.1155/2021/6548479

**Published:** 2021-10-13

**Authors:** Xuni He, Zhuhua Dai, Peina Shi, Jiemin Hong

**Affiliations:** Gastroenterology Department, Ningbo Yinzhou No. 2 Hospital, No. 998, Qianhe Road, Yinzhou District, Ningbo City, Zhejiang Province 315199, China

## Abstract

**Objective:**

Liver cirrhosis is a common, often progressive, and usually fatal disorder. Upper gastrointestinal bleeding is a leading cause of death in patients with liver cirrhosis. The purpose of this study was to evaluate the effectiveness of somatostatin combined with restricted fluid resuscitation in the treatment of upper gastrointestinal bleeding in the patients with liver cirrhosis.

**Methods:**

From January 2018 to December 2020, 84 patients with liver cirrhosis complicated by upper gastrointestinal bleeding admitted to the Department of Gastroenterology of Ningbo Yinzhou No. 2 Hospital were selected as study participants. They were randomly assigned into the study group (*n* = 42) and control group (*n* = 42). All patients were given intravenous drip of somatostatin. The study group was supplemented with restricted fluid resuscitation therapy. The hemoglobin (Hb), platelet, fibrinogen, hematocrit, transfusion volume of red blood cells, hemostatic time, hemostatic rates in 0 h–24 h, 24 h–48 h, and >48 h, rebleeding rates, resuscitation rate, and incidence rates of complications were compared between the two groups 48 h after treatment.

**Results:**

It was found that the Hb, platelet, fibrinogen, and hematocrit were notably increased in the study group compared to the control group 48 h after treatment (*P* < 0.01). The proportion of patients with excellent response was notably higher in the study group than in the control group (*P* < 0.05). The overall response rate of the study group was 90.48%, which was significantly higher than 71.43% in the control group (*P* < 0.05). The study group had lower transfusion volume of red blood cells, shorter hemostatic time, and lower rebleeding rates than the control group (*P* < 0.01). The hemostatic rate of 0 h–24 h in the study group was remarkably higher than that in the control group (*P* < 0.05). The hemostatic rate of >48 h in the study group was lower than that in the control group (*P* < 0.05). The overall incidence rate of complications in the study group was 9.52%, which was significantly lower than 30.95% in the control group (*P* < 0.05).

**Conclusion:**

These data suggest that intravenous drip of somatostatin followed by restricted fluid resuscitation leads to a better clinical efficacy in treating upper gastrointestinal bleeding in patients with liver cirrhosis considering higher resuscitation rate and hemostatic rate and reduced incidence of complications, which is conducive to the recovery of patients and worthy of further clinical promotion.

## 1. Introduction

Liver cirrhosis is one of the common severe diseases, which is mainly caused by connective tissue hyperplasia and nodular regeneration caused by diffuse liver injury. Clinical decompensation of liver cirrhosis is characterized by abdominal dropsy, septicemia, variceal bleeding, encephalopathy, and nonobstructive jaundice [1], which seriously affect the patient's life and health. Liver cirrhosis has been considered as an advanced liver disease that eventually leads to death in the absence of liver transplantation [2]. In developed countries, liver cirrhosis is the cause of increased incidence rate and mortality rate. It is regarded as the fourteenth most common cause of death in the world, but ranked fourth in central Europe. According to different stages of disease, the one-year mortality of liver cirrhosis varies from 1% to 57% [3].

At the end stage of disease, upper gastrointestinal bleeding is one of the most common complications of liver cirrhosis, which is mainly induced by esophageal and gastric varices and rupture of gastric varices [4]. Upper gastrointestinal bleeding is located near the Treitz ligament, with the mortality of 6%–10% [5]. It has been reported that the mortality of liver cirrhosis complicated with upper gastrointestinal bleeding exceeds 40.0%, which poses a great threat to the life and safety of patients [1]. Therefore, it is of great clinical significance to take early preventive and therapeutic measures to reduce the mortality. The treatment medicines such as nonselective *β-*receptor blockers, statins, oral antibiotics, and anticoagulants have been used in various combinations to prevent and treat complications of liver cirrhosis [6, 7]. Somatostatin and its analogues are a peptide hormone containing 14 amino acids isolated from the hypothalamus. It can increase the sensitivity of visceral vessels to vasoconstrictors, reduce portal vein pressure, block vasodilation, and promote visceral vasoconstriction [8]. Fluid resuscitation with colloidal and crystalline solutions is an effective method and a common intervention in acute medicine. Clinically, the selection of resuscitation fluid depends on physiological principles but largely varies from clinician to clinician [9]. It is the basis of nursing care for patients with sepsis, hemorrhagic shock, and other life-threatening diseases [10]. Restricted fluid resuscitation mainly refers to controlling the fluid input speed to ensure that the patient's blood pressure is maintained at a low and stable level, improve the body's self-protective compensation function, and finally achieve the best and maximum oxygenation and volume expansion with the minimum total amount of fluid [11].

Numerous studies have been conducted on the somatostatin alone for the treatment of bleeding in liver cirrhosis [12], esophageal varices [13], and upper gastrointestinal bleeding [14]. However, few studies have been found on the combination of somatostatin and fluid resuscitation in the treatment of liver cirrhosis and upper gastrointestinal bleeding. In this study, the application of somatostatin combined with restricted fluid resuscitation to 42 liver cirrhosis patients with upper gastrointestinal bleeding was analyzed, which might provide a theoretical basis for clinical treatment.

## 2. Materials and Methods

### 2.1. Study Design

From January 2018 to December 2020, 84 patients with liver cirrhosis complicated by upper gastrointestinal bleeding admitted to the Department of Gastroenterology of Ningbo Yinzhou No. 2 Hospital were selected as study participants. All patients were examined by liver function tests and transabdominal ultrasound, fulfilling the guidelines for the prevention and management of gastroesophageal varices and variceal hemorrhage in cirrhosis. All patients presented gastrointestinal bleeding symptoms such as hematemesis and black stool 24 hours before admission, with a blood volume of more than 1000 ml, accompanied by varying degrees of hemoglobin reduction and blood pressure reduction. These 84 patients were randomly assigned into the study group (*n* = 42) and control group (*n* = 42). This study has been approved by the Ethics Committee of Ningbo Yinzhou No. 2 Hospital.

### 2.2. Inclusion and Exclusion Criteria

All participants were diagnosed with liver cirrhosis and upper gastrointestinal bleeding through a variety of examinations, such as blood routine, gastroscopy, selective arteriography, CT, MRI, and color Doppler ultrasound. All patients and their families agreed to participate in the study, with a high degree of cooperation, with complete clinical data. Those who had any of the following conditions were excluded: administration of nonsteroidal, acid-inhibitory and anti-inflammatory drugs; severe organic diseases such as respiratory failure, heart failure, and cerebral infarction; upper gastrointestinal bleeding caused by noncirrhotic factors, such as gastrointestinal surgery and peptic ulcer; infectious disease; primary liver cancer; intolerance to gastroscopy; and mental or cognitive impairment.

### 2.3. Treatment Protocols

After admission, the two groups received regular care involving but not limited to fasting for 3 days, liver protection, antihypertensive drugs to portal vein, inhibition of gastric acid, and anti-infection. Blood transfusion was carried out on the patients if necessary. In the meantime, the vital signs of the patients were closely observed, and urination and defecation were recorded within 24 hours. The control group was given intravenous infusion of somatostatin (specification: 3 mg, National Permission No. H20066708, Yangzi River Pharmaceutical Group Co., Ltd., CN). First, somatostatin with 0.250 mg as the loading dose was intravenously injected into the patients, and then intravenous drip was performed immediately at the speed of 0.250 mg/h. The usage dose of somatostatin could be added to 0.375 mg/h or 0.500 mg/h according to the situation. In order to prevent rebleeding, intravenous administration of somatostatin was kept for 72 hours after the bleeding was controlled. The study group received somatostatin injection and restricted fluid resuscitation. In general, glucose injection was taken as main fluid and sodium injection was avoided except levofloxacin injection. The total volume of infusion was controlled within 1000 ml/24 h (not including blood transfusion: the maximum amount ≤400 ml/24 h). The infusion speed was controlled under 20–40 drops/min. The patients without obvious shock received infusion at the speed of 20 drops/min. Those patients with lower systolic blood pressure (<80 mmHg) received infusion at a higher dropping speed. However, the maximum dropping speed shall be controlled at ≤40 drops/min. During this period, the central venous pressure, arterial pressure, and urine volume of the patients should be closely observed.

### 2.4. Main Outcome Measures

All study participants were examined 48 h after treatment for their hemoglobin (Hb) (g/L), platelet (×10^9^/L), fibrinogen (g/L), and hematocrit (L/L). The transfusion volume of red blood cells (RBC), hemostatic time, hemostatic rates in 0 h–24 h, 24 h–48 h, and >48 h, rebleeding rates, resuscitation rate, and incidence rates of complications including hepatic encephalopathy, ascites, spontaneous peritonitis, hepatorenal syndrome, and hydrothorax were compared between the two groups. Hemostasis was used to reflect clinical efficacy and classified into excellent, good, and nonresponse: excellent response, the absence of hematemesis and gastrointestinal reactions including hematemesis and hematochezia, stable or increased Hb levels, stable blood pressure and heart rate, and clear or colorless gastric tube drainage fluids within 48 h after treatment; good response, the absence of hematemesis and gastrointestinal reactions, stable Hb levels, blood pressure, and heart rate, and clear or colorless gastric tube drainage fluids within 72 h after treatment; nonresponse, continues hematemesis and hematochezia, red and kermesinus gastric tube drainage fluids, continues reduction of Hb levels and blood pressure, and increased heart rate within 72 h after treatment. Overall response rate = (excellent response + good response)/cases × 100%.

### 2.5. Statistical Analysis

All data were processed by SPSS23.0 statistical software. The measurement data were expressed as a manner of mean ± standard deviation and compared using the *t*-test. The counting data were described by rate or ratio and compared using the chi-square test. *P* < 0.05 indicated the difference was statistically significant.

## 3. Results

### 3.1. Baseline Characteristics of Study Participants

The study group encompassed 26 males and 16 females, with an average age of 49.13 ± 8.23 years. According to Child–Pugh class of liver function, there were 3 cases evaluated as A class, 25 cases as B class, and 14 cases as C class (28 cases of hepatitis B-induced liver cirrhosis and 14 cases of alcoholic cirrhosis; 17 cases with gastric varices and 25 cases without). The control group included 29 males and 13 females, with an average age of 43.32 ± 8.21 years, and there were 2 cases of Child–Pugh A class, 27 cases of Child–Pugh B class, and 13 cases of Child–Pugh C class (26 cases of hepatitis B-induced liver cirrhosis and 16 cases of alcoholic cirrhosis; 20 cases with gastric varices and 22 cases without). These data between the two groups revealed no significant difference on age, gender, Child–Pugh class of liver function, causes of liver cirrhosis, and the presence of gastric varices (*P* > 0.05).

### 3.2. Clinical Efficacy of Intravenous Drip of Somatostatin Alone or Followed by Restricted Fluid Resuscitation

It was found that the Hb, platelet, fibrinogen, and hematocrit were notably increased in the study group compared to the control group 48 h after treatment (*P* < 0.01; Table 1). After treatment, the clinical efficacy of the two groups was improved. Excellent response was found in 28 patients, good response was found in 10 patients, and nonresponse was found in 4 patients in the study group. Excellent response was found in 18 patients, good response was found in 16 patients, and nonresponse was found in 8 patients in the control group. The proportion of patients with excellent response was notably higher in the study group than in the control group (*P* < 0.05). The proportions of patients with good response and nonresponse did not differ between the two groups. The overall response rate of the study group was 90.48%, which was significantly higher than 71.43% in the control group (*P* < 0.05; Table 2). There were 9 nonresponders in the control group, among which 5 cases were given endoscopic treatments, 2 cases were given surgical treatments, and 1 case died of hemorrhagic shock. There were 4 nonresponders in the study group, among which 3 cases were given endoscopic treatments, 1 case was given surgical treatments, and none died of hemorrhagic shock.

### 3.3. High Resuscitation Rate after Intravenous Drip of Somatostatin Alone or Followed by Restricted Fluid Resuscitation

As listed in Table 3, the resuscitation rate in the study group and the control group was 90.00% and 82.60%, respectively (*P* > 0.05). The infusion volume in the study group was significantly less than that in the control group (*P* < 0.05).

### 3.4. High Hemostatic Rate within 24 h after Intravenous Drip of Somatostatin Alone or Followed by Restricted Fluid Resuscitation

As shown in Table 4, the study group had lower transfusion volume of red blood cells, shorter hemostatic time, and lower rebleeding rates than the control group (*P* < 0.01). During the time of 0 h–24 h, 24 h–48 h, and >48 h, the cases, who succeeded in hemostasis, in the study group were 24 (57.14%), 13 (30.95%), and 5 (11.90%), respectively, and the cases in the control group were 15 (35.71%), 12 (28.57%), and 15 (35.71%), respectively. The hemostatic rate of 0 h–24 h in the study group was remarkably higher than that in the control group (*P* < 0.05). There was little difference between the hemostatic rate of 24 h–48 h in the study group and the control group (*P* > 0.05). The hemostasis rate of >48 h in the study group was lower than that in the control group (*P* < 0.05).

### 3.5. Intravenous Drip of Somatostatin Alone or Followed by Restricted Fluid Resuscitation Reduced the Incidence of Complications

After treatment, the patients in the two groups experienced different complications, such as hepatic encephalopathy, ascites, spontaneous peritonitis, hepatorenal syndrome, and hydrothorax. The overall incidence rate of complications in the study group was 9.52%, which was significantly lower than 30.95% in the control group (*P* < 0.05; Table 5).

## 4. Discussion

Liver cirrhosis is regarded as an advanced chronic liver disease with many complications, of which upper gastrointestinal bleeding is one of the most common acute and critical diseases [15]. Upper gastrointestinal bleeding is usually defined as bleeding near the Treitz ligament. It involves variceal and nonvariceal types. Variceal upper gastrointestinal bleeding is most frequently caused by gastroesophageal varices and isolated gastric varices. Nonvariceal upper gastrointestinal bleeding is caused by a series of factors, such as peptic ulcer, gastroduodenal erosion, erosive esophagitis, arteriovenous malformations, and upper gastrointestinal tumors [16, 17]. The main clinical manifestations of upper gastrointestinal bleeding are hematemesis (bright red emesis or coffee-ground emesis), hematochezia, hemorrhagic shock, and hemodynamic disorder. It might develop secondary symptoms, such as syncopation attacks, fatigue, and weakness. In severe cases, it will lead to acute peripheral circulation failure, incomplete perfusion of important organs, acute hypoxia, and ischemia of cells and finally induce hepatic encephalopathy and hepatic necrosis [18, 19]. It has been reported that upper gastrointestinal bleeding in the patients caused mortality ranges between 3% and 14%, which is associated with rebleeding [20]. Therefore, how to effectively control bleeding is the key to improve the survival rate and reduce the mortality.

With the continuous development of clinical research, the concept of restricted fluid resuscitation has been put forward. It mainly refers to controlling the infusion speed and volume to ensure that the patient's blood pressure is maintained at a relatively low and stable level, which finally achieves the best effect of hemostasis [21, 22]. The organ edema and organ dysfunction caused by excessive fluid infusion were reported in some clinical data [23, 24]. A small amount of fluid can avoid bleeding caused by diluting blood and filling blood vessels due to excessive amount of fluid. Restricted fluid resuscitation is associated with better outcomes, such as decreased incidence of complications and risk of death [25, 26]. In this study, the resuscitation rate of the study group was significantly higher than that of the control group. The hemostatic rate from 0 h to 24 h in the study group was significantly higher than that in the control group, and the rate after 48 h in the study group was remarkably lower than that in the control group. The data suggested that, for patients with upper gastrointestinal bleeding due to liver cirrhosis, somatostatin combined with restricted fluid resuscitation was associated with increased resuscitation rate and reduced mortality, which achieved the purpose of hemostasis in a short time. Duan et al. indicated that the patients with upper gastrointestinal bleeding, who received the combination of pantoprazole, somatostatin, and thrombin, revealed distinctly higher immediate hemostasis rate and hemostasis rate within 24 h [27]. The findings indirectly showed the less effectiveness in the treatment of somatostatin alone. In addition, Vincent et al. also suggested that fluid administration is a key intervention for hemodynamic resuscitation, which ensures the sufficient oxygen supply to important organs and reduces nephrotoxicity for the sepsis patients [28]. The present study demonstrated that the patients who received combination of somatostatin and restricted fluid resuscitation showed significantly higher overall response rate and lower incidence of complications, suggesting combination therapy can better improve the therapeutic effect and prognosis. These findings were similar to a previous study by Macdonald et al. which revealed that restricted fluid resuscitation increased survival of sepsis patients [21].

In conclusion, compared with somatostatin alone, the concurrent application of restricted fluid resuscitation and somatostatin is associated with better resuscitation rate, rapid hemostasis effect, and reduced incidence of complications, which is worthy of further clinical promotion. However, the limitations of small sample size and short observation time might lower the reliability of experimental data. Further study on large sample size and long observation time should be conducted in near future.

## Figures and Tables

**Table 1:** The Hb, platelet, fibrinogen, and hematocrit between the two groups.

Group	*n*	Hb (g/L)	Platelet (×10^9^/L)	Fibrinogen (g/L)	Hematocrit (L/L)
Control group	42	87.19 ± 9.71	79.94 ± 7.20	3.37 ± 0.57	41.40 ± 8.69
Study group	42	96.43 ± 11.03	88.86 ± 16.47	4.29 ± 0.54	47.04 ± 9.13
*P*		<0.01	<0.01	<0.01	<0.01

**Table 2:** The overall response rates between the two groups.

Group	*n*	Excellent response (*n*)	Good response (*n*)	Nonresponse (*n*)	Overall response rate (*n* (%))
Control group	42	18	16	8	30 (71.43)
Study group	42	28	10	4	38 (90.48)
*χ* ^2^	—	—	—	—	4.941
*P*	—	—	—	—	0.026

**Table 3:** Resuscitation rate and infusion volume between the two groups.

Group	*n*	Resuscitation	Death	Resuscitation rate (*n* (%))	Infusion volume (mL)
Control group	42	31	11	31 (73.81)	3177.27 ± 129.45
Study group	42	39	3	39 (92.86)	2021.50 ± 78.36
*χ* ^2^	—	—	—	5.486	34.563
*P*	—	—	—	0.019	<0.001

**Table 4:** Hemostatic rate between the two groups.

Group	RBC transfusion (U)	Hemostatic time (h)	Rebleeding (*n* (%))	0 h–24 h (*n* (%))	24 h–48 h (*n* (%))	>48 h (*n* (%))
Control group	3.14 ± 0.35	29.65 ± 5.78	14 (33.33%)	15 (35.71)	12 (28.57)	15 (35.71)
Study group	2.55 ± 0.43	23.89 ± 5.84	5 (11.90%)	24 (57.14)	13 (30.95)	5 (11.90)
*t*/*χ*^2^	6.896	4.543	2.347	3.877	0.057	6.563
*P*	<0.01	<0.01	0.019	0.049	0.811	0.010

**Table 5:** The incidence rate of complications between the two groups.

Group	Hepatic encephalopathy (*n* (%))	Ascites (*n* (%))	Spontaneous peritonitis (*n* (%))	Hepatorenal syndrome (*n* (%))	Hydrothorax (*n* (%))	Overall incidence (*n* (%))
Control group	5 (11.90)	3 (7.14)	2 (4.76)	2 (4.76)	1 (2.38)	13 (30.95)
Study group	1 (2.38)	1(2.38)	1(2.38)	1(2.38)	0 (0.00)	4 (9.52)
*χ* ^2^	—	—	—	—	—	5.974
*P*	—	—	—	—	—	0.015

## Data Availability

The data used to support the findings of this study are included within the article.
